The article "CNN-LSTM Hybrid Model for Kinematic Feature Analysis and Parabolic Radian Prediction in Basketball Videos" was retracted in 2023. Reasons: signs of a paper mill; suspected computer-generated content; unreliable results or conclusions; lack of ethics approval or compliance.

# CNN-LSTM Hybrid Model for Kinematic Feature Analysis and Parabolic Radian Prediction in Basketball Videos

**DOI:** 10.1155/2021/7844472

**Published:** 2021-09-23

**Authors:** Ji Rong, Yitong Chen, Jianxin Yang

**Affiliations:** School of Sports Training, Shenyang Sport University, Shenyang 110102, Liaoning, China

## Abstract

With the improvement of living standards around the world, people's love for sports has also increased; basketball is especially loved by people. It is of great importance to provide sound motor instruction for basketball. To this end, this paper comprehensively investigates the dependence between the optimal release conditions and the corresponding shooting arm movements in basketball players. We carry out kinematic feature analysis of basketball sports videos, propose a hybrid CNN-LSTM model that can predict the arc of the shooting parry, and identify the key movements of the arm joint that produce optimal release velocity, angle, and backspin in short-, mid-, and long-range shots. The experiment demonstrates that the model has three rigid planar links with rotational joints that mimic the shoulder, elbow, and wrist joints of the upper arm, forearm, and hand, which are better at guiding the optimal ball release speed, angle, and backspin for different players with the fastest ball speed being about 4.6 m/s and the slowest being about 1.7 m/s.

## 1. Introduction

With the improvement of the global standard of living, people's love for sports has also increased; in particular, basketball is loved by people. It is ornamental, for example, NBA, and athletic and is also an essential game for the Olympic Games. Thus, it is of great importance to provide reasonable sport instruction for basketball [1].

In basketball, a proper pitching arc can improve the hitting rate. Therefore, many studies have been conducted to analyze the kinematic characteristics in basketball sports videos [2, 3]. Good basketball players throw the ball with a nice arc, proper downward spin, and minimal lateral deviation from the optimal shooting plane. They manipulate their shoulders, elbows, and wrists to produce the best ball speed, angle, and angular velocity at release. Analyzing the kinematics of the shooting arm is critical to understand good shooting [4]. The study in [5] proposed six key teaching points for jump shots based on any basketball shooting studies and mentioned that photomechanical studies have not clearly identified the optimal coordination of human joint movements.

Several previous studies [6–8] measured shoulder, elbow, and wrist motion during a pitcher's jump shot and reported increased range effect. For free throws, the work in [9] represented the movements of shooting arm joints and investigated the techniques for high success rate shots. Their findings and measurements varied, as they investigated different shooting skills and situations. To our knowledge, no one has used a dynamic simulation model containing the ball and the shooter's arm to analyze the kinematics of basketball shooting. In wheelchair basketball, the work in [10] used a two-dimensional three-state simulation model to investigate the optimal release conditions for free throws and the corresponding arm movement patterns.

The article "CNN-LSTM Hybrid Model for Kinematic Feature Analysis and Parabolic Radian Prediction in Basketball Videos" was retracted in 2023. Reasons: signs of a paper mill; suspected computer-generated content; unreliable results or conclusions; lack of ethics approval or compliance.

There are also many programs that explore basketball movements to achieve kinematic feature analysis of basketball sports videos [11]. For example, traditional action recognition methods have static features based on shape and contour, and dynamic features based on optical flow and motion information. The study in [12] aims to achieve action recognition by doing shape matching of key video frames extracted from the video with the saved original action. The study in [13] computes the optical flow field of a target in a video using fuzzy optical flow features and achieves online action recognition by template matching. The study in [14] proposes expressing the action recognition of a target by features of key point motion history. The features extracted by traditional methods are manually designed features, and thus the performance of action recognition is not high.

In recent years, many action recognition methods based on deep learning have emerged. The study in [15] is an extension of the ordinary CNN to a 3D CNN with time series information. The network performs feature representation in the spatial and temporal dimensions of the video data, and the introduction of 3D convolutional kernels is more conducive to the analysis of the action information of the characters in the video. The P-CNN model proposed by [16] captures the action information of the person in the video by using a single frame of video data as well as optical flow information. The study in [17] is the most typical deep learning framework used, which is a deep dual-stream CNN combining spatial and temporal features, while proposing to use only the joint point portion of the human pose in the video for feature extraction from CNN. The study in [18] proposed the part-aware long short-term memory (LSTM) network, which mainly uses the collected skeletal data to achieve the analysis of human pose. In summary, the main idea of these deep learning methods is to capture the high-level semantic features of actions based on CNN models. However, it cannot guide or predict the action of a specific athlete's basketball shot.

We more fully investigate the dependence between the optimal release conditions and the corresponding short arm motion. In this paper, we perform kinematic feature analysis of basketball sports videos, propose a hybrid CNN-LSTM model that can predict the arc of the shooting parry, and identify the key movements of the arm joint that produce optimal release velocity, angle, and backspin in short-, mid-, and long-range shots.

The article "CNN-LSTM Hybrid Model for Kinematic Feature Analysis and Parabolic Radian Prediction in Basketball Videos" was retracted in 2023. Reasons: signs of a paper mill; suspected computer-generated content; unreliable results or conclusions; lack of ethics approval or compliance.

## 2. Related Technologies

### 2.1. LSTM

LSTM belongs to and is the optimization of recurrent neural networks (RNNs), whose main applications are in time series analysis and prediction [16, 19]. Its internal structure is more complex, and it is a more complex recurrent network structure of neurons through a unique gating unit to selectively transmit information [6, 20].

(1) $$\begin{array}{c} f_{t}=\sigma \left(W_{f}x_{t}+U_{f}h_{t-1}+b_{f}\right),\\ i_{t}=\sigma \left(W_{i}+U_{i}h_{t-1}+b_{i}\right),\\ {\tilde{C}}_{t}=\tanh\left(W_{c}x_{t}+U_{c}h_{t-1}+b_{c}\right),\\ C_{t}=f_{t}\times C_{t-1}+i_{t}\times \tilde{C},\\ O_{t}=\sigma \left(W_{o}x_{t}+U_{o}h_{t-1}+b_{o}\right),\\ h_{t}=O_{t}\times \;\tanh\left(C_{t}\right), \end{array}$$

where *x*_*t*_ is the input vector of the LSTM unit; *h*_*t*_ is the output vector of the LSTM unit; *W*, *U*, and *b* are the weight matrix and bias vector parameters; *σ* represents the Sigmoid [6] activation function; and tanh is the hyperbolic tangent function. In Figure 1, *i*_*t*_ represents the input gate, *O*_*t*_ represents the output gate, *f*_*t*_ represents the forgetting gate, and ${\tilde{C}}_{t}$ represents the memory gate. For the input and output gates, the corresponding weight of each gate is calculated and Sigmoid is taken as the activation function. Sigmoid takes the values within [0,1]. If the output value is 1, the corresponding value should be stored, but if it is 0, the corresponding value should be discarded completely. Tanh function in the memory gate is used to determine how much new information should be reflected in the cell state. Then, the previously calculated *i*_*t*_ and *C*_*t*_ values are added to the dot product of the values calculated by the forgetting gate, the previous cell state values, and the dot product of *i*_*t*_ to calculate the information to be reflected in *C*_*t*_. Finally, the value calculated by the output gate is obtained by multiplying the calculated unitary state value by tanh [16] to calculate the output value *h*_*t*_, and the output result is sent to the attention mechanism [21].

### 2.2. Attention Mechanisms

Attention is a well-known concept and a useful tool for deep learning. Neural networks with attention have been successful in machine translation [5], image cautioning [16], and speech recognition [21]. It is well known that RNN often has the problem of gradient disappearance because the time series is too long. LSTM can effectively solve this problem by capturing the dependencies of long time series more easily than RNN. However, it has been experimentally observed that in some cases, especially in very long sequences, the LSTM does not always remember long interdependencies and correlations correctly [13]. This leads to a decrease in the performance of the neural network with the passage of time, which leads to the so-called long-range dependence problem. Attention alleviates this problem by retaining all source input hidden state sequences at each time step and placing more attention and importance on the most relevant part of the sequence to produce the output.

The article "CNN-LSTM Hybrid Model for Kinematic Feature Analysis and Parabolic Radian Prediction in Basketball Videos" was retracted in 2023. Reasons: signs of a paper mill; suspected computer-generated content; unreliable results or conclusions; lack of ethics approval or compliance.

In order to better grasp the useful information in the new codes and to obtain significant spatiotemporal features, attention is introduced into our model. By assigning different attention probability weight, it follows with interest some trends or changes that occur in the training dataset and assigns more probability weight to enhance the newly encoded features. The mathematical formula for attention is as follows:

(2) $$\begin{array}{c} e_{ij}=\tanh\left(W_{1}h_{i}+W_{2}h_{j}+b_{\alpha }\right),\\ a_{ij}=\text{soft}\max\left(e_{ij}\right)=\frac{\exp\left(e_{ij}\right)}{\sum_{j}\exp\left(e_{ij}\right)},\\ H_{i}=\sum_{j}a_{ij}h_{j}, \end{array}$$

where *e*_*ij*_ denotes the relationship between *i*^th^ and *j*^th^ values, W is the weight, *b*_*α*_ is the bias, *a*_*ij*_ denotes the value of *i*^th^ attentional weight of the software function, and *H*_*i*_ denotes the final state of the output after passing attention. We use the above formula to calculate the corresponding weight of the new code in order to generate another new code with enhanced features.

### 2.3. CNN

CNN is an artificial neural network that has dominated in various computer vision tasks [13, 22, 23]. The key feature of the convolution operation is weight sharing: the kernel is shared over all image locations. Weight sharing creates the following features of the convolution operation: leaving the local feature patterns extracted by the kernel unchanged as the kernel moves over all image locations and detects the learned local patterns, learning the spatial hierarchy of feature patterns by downsampling combined with pooling operations to capture an increasingly larger field of view compared to a fully connected neural network, and improving the model by reducing the number of parameters to be learned efficiently [19, 24]. The pooling is commonly used in CNNs as a function of reducing the number of parameters and redundancy, and it can train weight and filters. One of the most typical pooling operations is max pooling. The fully connected layer forms the final one-dimensional output data and calculates its score according to the following formula:

(3) $$\begin{array}{c} y_{j}=\sum_{i=1}^{N}w_{i,j}x_{i}+b, \end{array}$$

where *y*_*j*_ is the output of the *j*^th^ neuron fully connected layer, *N* is the length of the input data, *w*_*i*,*j*_ denotes the neuron weight between the *i*^th^ input value and the *j*^th^ neuron, and *b* is bias. Once the results are calculated, the fully connected layer sends these values to higher-level connected units via an activation function to determine how much they contribute to the next prediction. The activation function is as follows:

(4) $$\begin{array}{c} \mu_{j}=g\left(y_{j}\right)=\max\left(0,y_{j}\right). \end{array}$$

*μ*_*j*_ is the output of the activation function. We use ReLU [17, 21] as the activation function, which can effectively prevent overfitting [16, 25]. Before outputting the final result, the dataset is sent to another activation function, called the linear activation function as follows:

(5) $$\begin{array}{c} \mu_{j}=f\left(y_{j}\right)=\mu_{j}. \end{array}$$

The article "CNN-LSTM Hybrid Model for Kinematic Feature Analysis and Parabolic Radian Prediction in Basketball Videos" was retracted in 2023. Reasons: signs of a paper mill; suspected computer-generated content; unreliable results or conclusions; lack of ethics approval or compliance.

## 3. Kinematic Model of Basketball Shooting

### 3.1. One-Handed Position Shots and Jump Shots

One-handed positioning and jump shots are most commonly used in modern basketball. The shooter holds the ball in his hand near his forehead, lifts and extends his elbow, and slams his wrist forward. The nonshooting arm helps support the ball and allows shots to be taken at the desired release position. Several previous studies have shown that the shooter should keep the ball, wrist, elbow, and shoulder in a plane perpendicular to the target [26]. The ball should be released with proper backspin and good arc and should not deviate from the optimal shot plane, including the target and ball release point.

### 3.2. Projectile Arm Geometry

We used a shot arm model similar to the two-dimensional three-section model of [27]. It is assumed that the shooting arm moves in the vertical plane and has three rigid linkages, where the upper arm, forearm, and hand have rotational joints, as well as shoulder, elbow, and wrist joints. The coordinate system of the shooting arm and the basketball is shown in Figure 2.

Before the ball touches the basket or rim, the center of the ball moves in the plane of the angular velocity vector of the ball and the connecting rod perpendicular to the plane of the initial stroke path [18, 28].

Subject *B* and the point *B*^*∗*^ denote the basketball and the center of the ball. The lengths of the upper arm, forearm, hand, and ball radius were *L*_*U*_, *L*_*F*_, *L*_*H*_, and *R*_*b*_, respectively. The position of the fingertips can be written using the following angles: Ψ_*S*_ from the horizontal plane to the upper arm linkage, Ψ_*E*_ from the upper arm to the forearm linkage, and Ψ_*W*_ from the forearm to the hand linkage. The unit vectors *I*, *J*, and *K* are attached to the ground. The *JK* plane is vertical, and the *K* vector is up. The other unit vectors are attached to the linkage and the ball as shown in Figure 2.

The article "CNN-LSTM Hybrid Model for Kinematic Feature Analysis and Parabolic Radian Prediction in Basketball Videos" was retracted in 2023. Reasons: signs of a paper mill; suspected computer-generated content; unreliable results or conclusions; lack of ethics approval or compliance.

### 3.3. Shooting Arm Kinematics

We consider the position and orientation of the triple linkage plane arm of the lens. The relationship between joint angle and fingertip velocity is derived. The horizontal and vertical components of the fingertip velocity with respect to the shoulder joint (assumed to be fixed) can be expressed as

(6) vNH^/S·J=−Ψ˙SLUsin  ΨS−Ψ˙S+Ψ˙ELFsinΨS+ΨE−Ψ˙S+Ψ˙E+Ψ˙WLHsinΨS+ΨE+ΨW,vH/S·K=Ψ˙SLUcos  ΨS+Ψ˙S+Ψ˙ELFcosΨS+ΨE+Ψ˙S+Ψ˙E+Ψ˙WLHcosΨS+ΨE+ΨW.

The surface velocity of the ball at fingertip contact point $\hat{B}$ can be described as

(7) vNB^=vNB∗+ω×RbjB,

where ^*N*^**v**^*B*^*∗*^^ is the velocity at the center of the ball, *ω* is the angular velocity of the ball, and **j**_*B*_ is the unit vector from the fingertip to the center of the ball. When the release is ^*N*^**v**^*B*^ equal to ^*N*^**v**^*H*^, the ball leaves the fingertip and does not slide between the fingertip and the ball surface, and the angular velocity of the ball can be written as $\omega \cdot I={\dot{\Psi }}_{S}+{\dot{\Psi }}_{E}+{\dot{\Psi }}_{W}+{\dot{\Psi }}_{B}$, where ${\dot{\Psi }}_{B}$ is the angle between the hand linkage and the line that includes the fingertip and the center of the ball.

### 3.4. Joint Angular Displacement of the Launch Arm at Release

Several previous studies have measured the joint angles of the shoulder, elbow, and wrist during the release of athletes during jump shots and free throws [28]. The study in [29] shows a jumping action in which the angle between the upper arm and the horizontal plane is about 51 degrees, the angle between the hand and the forearm is about 180 degrees, and the angle between the forearm and the horizontal plane at release is about 80 degrees. The study in [30] shows a graphical representation of a wooden stick to shooting motion, where the angle between the forearm and the horizontal plane is about 90 degrees and the angle between the forearm and the hand is 173 degrees to 201 degrees [31]. The study in [32] shows that the measured upper arm angles range from 28 to 38 degrees horizontally, with an average angle between the upper arm and forearm of about 135 degrees and an average wrist angle at release of about 190 degrees.

The article "CNN-LSTM Hybrid Model for Kinematic Feature Analysis and Parabolic Radian Prediction in Basketball Videos" was retracted in 2023. Reasons: signs of a paper mill; suspected computer-generated content; unreliable results or conclusions; lack of ethics approval or compliance.

We estimated possible release joint angles based on previous studies of short-range (horizontal distance *l* = 2 m from the center of the basket and vertical distance *h* = 0.05 m from the center of the basket), medium-range (*l* = 4 m, *h* = 0.15 m), and long-range (*l* = 7 m, *h* = 0.30 m) shot locations. Figure 1 shows an example set of shoulder, elbow, and wrist angles with LU = 3.0 m, LF = 3.0 m, and LH = 2.0 m for long-range shots when the ball release position and shoulder position are given. The angle of the shoulder joint with the horizontal plane ranges from 45 degrees (when the forearm and wrist joint is vertical) to 59 degrees (when the elbow angle is close to 18 degrees at 0). The manual linkage is located in a straight line, including the center of the ball at release [17, 33].

### 3.5. CNN-LSTM Model

The study in [34] found that video streaming data has a spatiotemporal correlation feature, which makes the video streams between connected regions influence each other. While increasing the spatiotemporal feature extraction of video stream sequences, this paper proposes to enhance the robustness and convergence of the CNN-LSTM prediction model using the RAdam optimization algorithm [24], which reduces the prediction error of the proposed model while reducing the model training time, and finally obtains a good prediction accuracy [35]. The model designed in this paper is shown in Figure 3.

The model process constructed in this paper includes data preprocessing, including removing outlier values, linear interpolation, and data normalization processing. The preprocessed basketball video data are input to the LSTM model, and a series of new sequences are generated with basketball video sequences of specific width as input and output. New data sequences are sent to the attention mechanism to enhance temporal features. The CNN model extracts the spatial feature output data from the image, reduces the parameters, and implements the redundancy function by passing them to the maximum pooling layer. Finally, the data are sent through the fully connected layer and linear activation function to the last hidden layer to produce the final prediction output.

In this study, the improved CNN-LSTM model is implemented with the following processing steps:

*Step 1*. The input historical video stream data is first constructed to contain the video stream spatiotemporal correlation feature matrix *X*, defined as
  (8) $$\begin{array}{c} X=\left[\begin{array}{ccccc} x_{1}^{1} & x_{2}^{1} & x_{3}^{1} & \cdots & x_{t-m}^{1}\\ x_{1}^{2} & x_{2}^{2} & x_{3}^{2} & \cdots & x_{t-m}^{2}\\ x_{1}^{3} & x_{2}^{3} & x_{3}^{3} & \cdots & x_{t-m}^{3}\\ \vdots & \vdots & \vdots & \cdots & \vdots \\ x_{1}^{i} & x_{2}^{i} & x_{3}^{i} & \cdots & x_{t-m}^{i} \end{array}\right], \end{array}$$
where *x*_*t*−*m*_^*i*^ is the basketball video frames collected at location *i* at time *t* − *m*, and *x*=(*x*_1_^*i*^, *x*_2_^*i*^, *x*_3_^*i*^,…, *x*_*t*−*m*_^*i*^) is the historical data traffic collected at location *i*.
*Step 2.* Input the feature matrix *X* to the multilayer CNN, extract the spatial features of the video stream data, and get the video stream sequence feature vector.
*Step 3.* Input the feature vectors to a multilayer LSTM network to extract time-dependent features.
*Step 4*. After completing the construction of the model network structure, the dropout layer [26, 36] is introduced and the RAdam optimization algorithm is applied to the training process in order to prevent overfitting of the data and long training convergence time. RAdam optimization algorithm is described in Algorithm 1.
*Step 5*. After the model is trained and tested, the final output of the predicted video stream sequence is described as
  (9) $$\begin{array}{c} h=\left\{h_{t-\left(m-1\right)},h_{t-\left(m-2\right)},h_{t-\left(m-3\right)},\ldots ,h_{t}\right\}, \end{array}$$
  where *h*_*t*_ is the predicted video traffic at time *t*, and *h* is the predicted video traffic sequence.

The article "CNN-LSTM Hybrid Model for Kinematic Feature Analysis and Parabolic Radian Prediction in Basketball Videos" was retracted in 2023. Reasons: signs of a paper mill; suspected computer-generated content; unreliable results or conclusions; lack of ethics approval or compliance.

## 4. Results and Analysis

### 4.1. Striding Jump Shot Technical Movement

Time-phase division is an important part of the study of technical movements, which are conducive to a more detailed and in-depth study of movement structure [5]. In the past, the temporal division of the action structure was mostly based on the sequence of activities of the action structure or the force during the action [17], but in this paper the temporal division of the stride jumping action is based on the combination of the action of the feet and the ground and the sequence of joint activities in the whole technical action. In order to determine the structure of the action and to facilitate the division of the time phase, combined with the filmed basketball video, we first determined the characteristic images of the stride jump shooting action; that is, based on the action of the feet and the ground and the sequence of joint activities, the critical points of different actions can be determined as follows: the moment of the left foot heel landing, the moment of the right foot leaving the ground and the right leg swinging forward, the moment of the arms raising the ball, the moment of the right foot landing and bending the knee to cushion, the moment of the hip and knee joint extension, the moment of jumping, the moment when both feet leave the ground, and the moment when both feet land on the ground to buffer 7 characteristic pictures. Accordingly, the whole action process of the stride jump shot is divided into 6 phases, namely, the left foot landing and braking phase, the right leg swinging forward phase, the ball lifting phase, the jumping phase, the vacant shot phase, and the landing cushion phase, as shown in Figure 4.

The article "CNN-LSTM Hybrid Model for Kinematic Feature Analysis and Parabolic Radian Prediction in Basketball Videos" was retracted in 2023. Reasons: signs of a paper mill; suspected computer-generated content; unreliable results or conclusions; lack of ethics approval or compliance.

Figure 4(a) shows the elastic potential energy stored for the jump from the moment of landing on the heel of the left foot to the moment of landing on the whole left foot all together.

Figure 4(b) shows the time from the moment the right foot leaves the ground to the moment the right foot hits the ground again.

Figure 4(c) shows that the ball is lifted from the flexion of the elbow joint to the relative fixation of the shoulder joint, at which time the ball is lifted from the flexion of the elbow joint to the lifting of the arms with the extension of the shoulder joint, and the range of the ball is significantly increased.

Figure 4(d) shows the time from the moment of the beginning of hip extension to the moment when the feet are about to step off the ground.

Figure 4(e) shows the time when the ball leaves the hand from the moment the feet leave the ground. During this phase, the lower limb joints are gradually extended as the body weight rises and the right upper limb, which is the shooting arm, completes the elbow extension and wrist shake before the body rises to the highest point.

Figure 4(f) shows the time from the moment the body starts to fall from the highest point to the moment the feet hit the ground.

### 4.2. Kinematic Characteristics of the Striding Jump Shot Technique

By dividing the temporal phases of the six action phases of the stride jump shot, the shooting action based on the landing cushion phase is over; therefore, only the first five technical phases are studied in this paper.

#### 4.2.1. Temporal Characteristics of the Straddle Jump Shot Technique

The time characteristics of each action phase of the stride jump shot technique are shown in Table 1. Through the analysis of the data, we can learn that the time spent in the whole action process is the longest in the air shot phase, followed by the ball lifting phase, followed by the right leg swing and jump, and the shortest in the left foot landing phase. The time consuming situation of each movement phase has a certain influence on the completion quality of the whole technical movement. The braking method after the left foot landing is the transition from the heel to the whole foot, and the shortest duration of the left foot landing phase is determined by this particular form of action; the longest duration of the jumping phase is due to the fact that, at the beginning of the jumping action, the torso is first extended, and this action causes small lowering of the body's center of gravity again and also increases the cushioning amplitude of the lower limbs, which in turn increases the duration of the lower limb stirring. The time spent in the right leg swing phase is mainly influenced by the change in the swing of the right leg and the different landing distances of the right foot; the time spent in the air shot phase is mainly influenced by the height of the jump and the time of the shot; the longer time spent in the ball lifting phase is due to the fact that the ball lifting action starts before the right leg swing hits the ground, runs through the whole jumping process, and ends when the body just enters the air state. In terms of the combined form of the stride jump shot technique, the technique can be seen as a combination of stride action and in situ jump shot action. Therefore, the characteristics of the time spent in each phase of the action can also reflect the coherence of the articulation between the stride action and the in situ jump shot action.

The article "CNN-LSTM Hybrid Model for Kinematic Feature Analysis and Parabolic Radian Prediction in Basketball Videos" was retracted in 2023. Reasons: signs of a paper mill; suspected computer-generated content; unreliable results or conclusions; lack of ethics approval or compliance.

#### 4.2.2. Technical Characteristics of Each Phase of the Stride Jump Shot

1. In the take-off stage of the left foot, at this time, the right foot has not left the ground, and the reaction force is pushed forward by the body and the right foot. After the right foot is pushed on the ground, the left foot quickly leaves the ground, and the left foot landing is conducive to maintaining body balance in the process of rapid forward movement.
2. Through the analysis of the basketball video and data, the characteristics of the left lower limb joint angles of the athletes when landing on the left foot were derived, as shown in Table 2. Analysis shows that the angle of the ankle joint is between 104°and 118°, the angle of the knee joint is between 126° and 161°, and the angle of the hip joint is between 112°and 146°; the different angles of the three joints reflect the different postures of the left lower limb when the athlete lands on the left foot. The angular characteristics of the knee joint indicate that the athlete's body center of gravity is lowered to different degrees with the landing of the left foot, but the lowering of the center of gravity is not uniform: the lowering of the body center of gravity is conducive to the rapid forward movement of the athlete's body to complete the braking of the left foot quickly. The different angular characteristics of the hip joint show that the athlete's torso has different degrees of forward leaning and the change of torso posture at this time is mainly to maintain their balance in the state of rapid forward movement of the body.
3. The right leg forward swing phase is from the moment the right foot leaves the ground to the moment the foot is fully on the ground again. According to the change of swinging posture of the right leg in the process of forward swing, it can be divided into two different postures, “knee flexion” and “knee extension”; the change of posture of the right leg in this stage is not only beneficial to the balance maintenance of the body in the state of single support of the left foot, but also beneficial to the right foot rapid braking on the ground.
4. Combining the analysis of the basketball video and the data in Table 3, we know that the joint angle of the right leg in the front swing basically shows that the values of the hip joint are larger than those of the ankle joint and knee joint; the reason is that the right lower limb stirs off the ground in the front swing by the right foot stomping when the ground reaction force has a certain speed, and stirs off the ground by the right hip flexion effect but also increases the swing speed of the right lower limb. The different angular characteristics of the hip joint reflect the difference of the athlete's hip extension, and on the other hand, they can also reflect the difference of the right lower limb stirrups of the ground by the ground reaction force. The intrinsic angular characteristics of the knee joint reflect the different folding positions of the upper and lower legs, and the angle of the ankle joint reflects the different degrees of flexion of the athlete's foot after stirring off the ground. In the early stage of the right leg swing, the right hip joint is flexed forward, the lower leg is gradually folded with the thigh under the influence of the knee flexion, and the hip joint is used as the power joint to accelerate; in the later stage of the swing, as the amplitude of hip flexion gradually decreases, the lower limb is gradually extended under the influence of the knee extension, and the ankle joint is gradually bent and flexed to prepare for the landing action. The change in the pendulum posture of the leg during the forward swing not only helps to maintain the body balance in the single-legged support state, but also enables the right foot to quickly land and brake to form a stable double-legged support.
5. The ball lifting phase starts before the right foot hits the ground, but the ball lifting action is mainly based on the flexion of the elbow joints; after the right foot hits the ground and brakes, the ball lifting action gradually changes from the flexion of the elbow to the lifting of both shoulder joints as the axis, and the amplitude of the ball lifting is obviously accelerated. After the body enters the air state, with the lowering of the body lift, the amplitude of the ball lifting with both shoulder joints decreases significantly, the body is fixed, and the ball lifting action ends at this point.
6. Figure 5 shows that the ball speed of the athletes in this phase varied, with the fastest ball speed being about 4.6 m/s and the slowest being about 1.7 m/s. The difference in ball speed not only reflects the inconsistency in the amplitude of the ball lifted by the athletes, but also reflects the difference in the amplitude of the upper limb movement. The analysis of the basketball video and the data in Table 4 showed that the degree of elbow flexion of both arms was different during the ball lifting phase, mainly because the elbow flexion was more pronounced in the arm of the shooter, the wrist of the dominant shooter produced an outward rotation of the palm with the ball lifting motion during the arm lifting process, and the joints of the right arm were higher than those of the left arm in the final stable shooting position. The position of each joint of the right arm is higher than that of the left arm in the final stable shooting position.
7. Jumping phase: Jumping is the process of the distal link as a fixed kind of explosive muscle exertion. After the right foot landing, the stride action ends and the body's center of gravity is lowered again with the landing of the right foot. The lowering of the body's center of gravity not only is conducive to increasing the stretching amplitude of the leg muscles, but also increases the force between the feet and the ground, which is more conducive to the jumping phase of the feet and the rapid extension of the lower limb joints.
8. Combining the basketball video and the data in Table 5, we know that, when jumping, the lower limb ankle, knee, and hip joints move in a different order. The hip joint is the first to extend under the role of arm lift. The extension of the hip joint enables the trunk and lower limbs to stay in the same vertical plane as much as possible when jumping, so that the body can use the vertical speed more effectively. At this time, the angle difference of the internal hip joint is reflected in the different inclination degrees of the human body when jumping. The greater the difference in trunk inclination, the worse the athlete's jumping ability. For example, the inclination of the trunk of athletes No. 3 and No. 7 is as high as 20 degrees. This posture is not only not conducive to the difficulty of the athlete in the jumping process, but also unfavorable to the body. The difference in the angle of the ankle joint in this stage was manifested in the external action in the form of the different power sequence of the ankle joint during the jump, in which the difference between no. 4 and no. 6 was the most significant, mainly due to the inconsistent extension of the ankle joint caused by the difference in the landing of the feet. The angle difference at the knee joint reflects the different degrees of passive stretching of the leg muscles after landing on one hand, and the stirrups and extensions of the lower limbs during the jump are not carried out simultaneously on the other. In the analysis of the video of the jumping phase, it was found that, with the extension of the hip and knee joints, the feet left the ground from the heel first and gradually transitions to the forefoot and finally the forefeet of both feet stomped off the ground.
9. After the feet leave the ground, the hip, knee, and ankle joints are fully flexed and extended as the center of gravity gradually rises, and the shoulder joints form a relatively stable state as the body rises and slows down. On the other hand, this helps to maintain the stability of the shooting arm's posture as it rises with the body.

The article "CNN-LSTM Hybrid Model for Kinematic Feature Analysis and Parabolic Radian Prediction in Basketball Videos" was retracted in 2023. Reasons: signs of a paper mill; suspected computer-generated content; unreliable results or conclusions; lack of ethics approval or compliance.

The shot exit time is cited at different moments before the body rises to the highest point, and in the vacant exit phase, the shot exit time has an impact on the quality of the completion of the entire shooting technique movement. The analysis of the video of the athlete's vacated spot phase shows that, in the stride jump shot technique, the shooting shot is completed at different moments before the athlete's body rises to the highest point. By analyzing the speed of the ball before and after it leaves the hand in Figure 6, we can learn that the speed increases to different degrees after the ball leaves the hand, and the change of the ball speed after leaving the hand is mainly influenced by the hand action, which is because the hand, as the end link of the shooting arm, has an important influence on the speed of the ball, the force of the ball, and the trajectory of the ball running in the air.

### 4.3. Pitching Arc Analysis Discussion

The angular velocity combinations of the shoulder, elbow, and wrist joints are plotted in each group shown in Figure 1 to produce optimal ball release velocity, angle, and backspin at 4.58 m/s, 47.5°, and 2*π* rad/s for short distances; 6.62 m/s, 46.0°, and 4*π* rad/s for medium distances; and 9.04 m/s, 46.0°, and 6*π* rad/s for long distances [16, 30]. When the shoulder velocity SN *v* is zero, there is no sliding between the fingertip and the ball surface at release. Reasonable conditions are ${\dot{\Psi }}_{S}>0$ (the vertical component of the elbow velocity is usually positive) and ${\dot{\Psi }}_{S}+{\dot{\Psi }}_{S}+{\dot{\Psi }}_{E}<{\dot{\Psi }}_{S}+{\dot{\Psi }}_{E}<0$ (the angular velocities of the forearm and hand are usually negative, and the magnitude of the angular velocity of the hand is greater than that of the forearm) used for calculation.

The article "CNN-LSTM Hybrid Model for Kinematic Feature Analysis and Parabolic Radian Prediction in Basketball Videos" was retracted in 2023. Reasons: signs of a paper mill; suspected computer-generated content; unreliable results or conclusions; lack of ethics approval or compliance.

Figure 7 shows the set of angular velocities of the shoulder, elbow, and wrist joints for optimal release conditions in shoulder-elbow-wrist angular velocity space. Figures 8(a) and 8(b) show the top and side views of the angular velocity group in Figure 8. Each line is a function of ${\dot{\Psi }}_{S}$, ${\dot{\Psi }}_{S}+{\dot{\Psi }}_{E}$ and ${\dot{\Psi }}_{S}+{\dot{\Psi }}_{E}<{\dot{\Psi }}_{W}$ functions.

For Ψ_*S*_+Ψ_*E*_=90° and Ψ_*W*_=0 (where the forearm and hand are vertical) for release, the vertical component of fingertip velocity is a function of ${\;\dot{\Psi }}_{S}$, but neither a function of ${\dot{\Psi }}_{S}+{\dot{\Psi }}_{E}$ nor a function of ${\dot{\Psi }}_{S}+{\dot{\Psi }}_{E}+{\dot{\Psi }}_{W}$. For short-, medium-, and long-range shots, the angular velocity of the shoulder can be calculated as ${\dot{\Psi }}_{S}$ = 15 9.22.4 and 30.7 rad/s. The shoulder rotation contributes to the vertical component of the ball velocity and is important for a good arc of the ball trajectory.

Several previous studies have measured the angular velocity of the shoulder, elbow, and wrist joints during release of shooters. Miller and Bartlett [37] denote the angular velocity of the arm joint to produce three different ball release velocities. As the ball release velocity increased, the magnitude of the elbow angular velocity increased, while the magnitude of the wrist angular velocity decreased, and there was almost no difference in the magnitude of the shoulder angular velocity for the three ball release velocities. Our kinematic analysis revealed possible combinations of angular velocities of the shoulder, elbow, and wrist joints. This may be one of the reasons for the different results of previous measurements of shooting arm motion.

Figure 9 shows the angular velocity combinations for mid-range releases with different backspin: 2*π*, 4*π*, and 6*π* rad/s. For releases Ψ_*S*_+Ψ_*E*_=90° and Ψ_*W*_=0 (where both forearm and hand are vertical), shoulder rotation contributes to the vertical component of the ball release velocity, and elbow and wrist rotation mainly affect backspin.

## 5. Conclusions

This study comprehensively investigates the dependence between the optimal release conditions and the corresponding shooting arm movements in basketball players. In this paper, we conduct kinematic feature analysis of basketball sports videos; e.g., a two-dimensional kinematic model of the shooter's arm is derived, including basketball used for short-range, mid-range, and long-range shots. The kinematic model estimates the angle and angular velocity of the shoulder, elbow, and wrist for a given set of ball release velocities, angles, and backspin. For each release condition, many combinations of shoulder, elbow, and wrist joint angular velocities with the fastest ball speed being about 4.6 m/s and the slowest being about 1.7 m/s are demonstrated. We also propose a hybrid CNN-LSTM model that predicts the arc of the shot and identify the key movements of the arm joint that produce the optimal release velocity, angle, and backspin in the short-, mid-, and long-range shots.

The article "CNN-LSTM Hybrid Model for Kinematic Feature Analysis and Parabolic Radian Prediction in Basketball Videos" was retracted in 2023. Reasons: signs of a paper mill; suspected computer-generated content; unreliable results or conclusions; lack of ethics approval or compliance.

Using previous research and our results, we found that shooters have a wide range of angular velocities in their arm joints to produce the ball release conditions they desire.

## Figures and Tables

**Figure 1:** Shoulder, elbow, and wrist joint groups during relaxation.

**Figure 2:** Geometry of the shooting arm with basketball.

**Figure 3:** Flow chart of the CNN-LSTM model with fused attention mechanism.

**Figure 4:** Time-phase division of the phase of the stride jump shooting action (a–f).

**Figure 5:** Characteristics of ball speed during the lifting phase of the player.

**Figure 6:** Characteristics of the ball speed before and after the player's shot in the air phase.

**Figure 7:** Angular velocity combinations of the upper arm, forearm, and hand at release during short-, medium-, and long-range shooting.

**Figure 8:** Relationship between joint angular velocities for short-, medium-, and long-range release: (a) forearm angular velocity vs. wrist angular velocity; (b) wrist angular velocity vs. shoulder angular velocity.

**Figure 9:** Relationship between joint angular velocities for mid-range release with 1, 2, and 3 Hz backspin: (a) forearm angular velocity vs. wrist angular velocity; (b) wrist angular velocity vs. shoulder angular velocity.

**Algorithm 1:** RAdam-based optimization algorithm.

**Table 1:** Time of each movement phase of the striding jump shot technique.

Stage	Left foot landing	Right foot forward swing	Takeoff	Empty hand	Landing buffer
Time/s	0.04±0.01	0.20±0.03	0.26±0.05	0.17±0.03	0.24±0.08

**Table 2:** Characteristics of lower limb joint degree when the left foot landed, in 8 athletes.

	1	2	3	4	5	6	7	8
Ankle angle	118.83	118.97	105.52	104.50	108.53	104.14	106.67	107.73
Knee angle	150.16	152.60	129.60	156.14	160.61	139.05	162.73	125.77
Hip angle	124.83	138.22	146.06	142.91	141.91	117.31	142.05	112.37

**Table 3:** Characteristics of joint angles during the right leg forward swing of the athlete.

	1	2	3	4	5	6	7	8
Ankle angle	109.07	106.60	113.85	106.63	103.22	91.93	107.23	100.17
Knee angle	91.77	91.44	102.23	98.87	89.29	97.96	103.56	104.62
Hip angle	103.29	134.99	120.24	109.33	97.54	130.78	123.90	126.17

The article "CNN-LSTM Hybrid Model for Kinematic Feature Analysis and Parabolic Radian Prediction in Basketball Videos" was retracted in 2023. Reasons: signs of a paper mill; suspected computer-generated content; unreliable results or conclusions; lack of ethics approval or compliance.

**Table 4:** Characteristics of upper limb joint angles during the ball lifting phase of the athlete.

	1	2	3	4	5	6	7	8
Right elbow angle	77.55	82.31	80.89	85.03	97.72	83.32	95.54	87.67
Left elbow angle	92.39	85.52	101.38	113.12	111.10	104.06	103.45	103.91
Diff.	14.84	2.21	20.49	28.09	13.38	20.74	7.91	16.24
Right shoulder angle	75.60	76.76	76.19	82.80	76.11	96.87	66.19	105.43
Left shoulder angle	82.08	80.05	87.78	95.43	91.55	98.20	78.76	98.95
Diff.	6.48	3.29	11.59	12.63	15.44	1.33	12.57	6.48

**Table 5:** Characteristics of lower limb joint angles during jumping of 8 athletes.

	Ankle joint			Knee joint			Hip joint		
	Left	Right	Diff.	Left	Right	Diff.	Left	Right	Diff.
1	123.32	116.50	6.82	137.29	142.58	5.29	148.77	154.32	5.55
2	120.71	121.81	1.10	127.78	142.15	15.37	154.84	162.91	8.07
3	121.11	101.21	19.90	124.19	133.75	9.56	164.26	143.84	20.42
4	140.85	108.85	32.30	124.43	140.01	15.58	143.26	139.66	3.60
5	102.80	98.84	3.96	115.15	112.96	2.19	117.91	132.45	14.54
6	134.36	113.66	20.70	124.99	144.41	19.42	144.13	141.06	3.07
7	101.78	113.55	1.97	132.80	109.66	23.14	134.78	161.33	26.55
8	104.48	99.61	5.87	125.60	118.19	7.51	119.52	129.51	9.99

## Data Availability

The dataset used in this paper are available from the corresponding author upon request.
